# Inhibition of lncRNA H19/miR-370-3p pathway mitigates neuronal apoptosis in an *in vitro* model of spinal cord injury (SCI)

**DOI:** 10.1515/tnsci-2021-0013

**Published:** 2021-03-01

**Authors:** Xin Li, Yan Qian, Kaihua Tang, Yang Li, Rui Tao, Chunyan Gong, Li Huang, Kaiwen Zou, Lindong Liu

**Affiliations:** Department of Rehabilitation Medicine, Qujing No. 1 Hospital, Yuanlin No. 1 Road, Qilin District, Qujing 655000, Yunnan, China

**Keywords:** SCI, lncRNA H19, miR-370-3p, NF-κB pathway

## Abstract

**Background:**

Spinal cord injury (SCI) is the most serious complication of spinal injury, often leading to severe dysfunction of the limbs below the injured segment. Conventional therapy approaches are becoming less and less effective, and gene therapy is a new research direction by now.

**Methods:**

The Sprague-Dawley rats were haphazardly assigned to two groups, namely sham group and SCI model group, and lncRNA H19 and miR-370-3p levels were investigated using reverse transcription-quantitative polymerase chain reaction (RT-qPCR). Correlation between lncRNA H19 and miR-370-3p was ascertained by luciferase report assay and RT-qPCR. After transfection with si-H19, miR-370-3p inhibitor, negative controls (NC), or both, primary spinal neurons were subjected to the simulation of lipopolysaccharide (LPS) for inducing *in vitro* model of SCI. Cell viability, apoptotic rate, caspase-3 activity, Bax and Bcl-2 protein, ROS generation, TNF-α, IL-1β, and IL-6 protein, as well as IκBα and p65 phosphorylation ratio were evaluated adopting 3-(4,5-dimethylthiazol-2-yl)-2,5-diphenyltetrazolium bromide (MTT), apoptosis, caspase-3 activity, ROS generation, and western blot assays, thereby searching for the specific action mechanism on LPS-induced spinal never injury.

**Results:**

SCI resulted in lncRNA H19 higher expression and miR-370-3p lower expression. LPS simulation raised a series of cellular biological changes, such as decreased viability, promoted apoptosis, generated ROS, and released inflammatory factors. lncRNA H19 inhibition reversed above LPS-induced changes. Besides, as the downstream target of lncRNA H19, miR-370-3p was oppositely regulated by lncRNA H19. The above biological changes induced by lncRNA H19 inhibition were reversed by miR-370-3p upregulation. Moreover, lncRNA H19 inhibition could block NF-κB pathway through miR-370-3p upregulation.

**Conclusion:**

Inhibition of lncRNA H19/miR-370-3p mitigated spinal neuron apoptosis in an *in vitro* model of SCI. This provided the possibility for clinical use of gene therapy.

## 1 Introduction

With the development of economy worldwide, the incidence rate of spinal cord injury (SCI) shows an annual increasing trend. According to statistics, there is about 10.4–83 million SCI cases suffering every year globally [1]. SCI is the most complication of spinal injury, which often leads to severe dysfunction of the limb below the injured segment, accompanied by sensory disturbance, spinal shock, motor dysfunction, autonomic nervous dysfunction, abnormal reflexes, and bladder dysfunction [2]. Once suffering from SCI, people maintain worse life standard with lower income. The treatment of SCI is always a big challenge in clinical application for doctors and scientists [3]. According to the degree of severity of SCI, the universal treatment approaches including drug therapy and surgery. At present, conventional drug therapy and surgery are becoming less and less effective especially for serious patients, and gene therapy become a new and hot research direction, especially non-coding RNAs (ncRNAs).

Long ncRNAs (lncRNAs) are a category of ncRNAs that possess the length of greater than 200 nucleotides [4,5]. Consistent with mRNA, lncRNA can exercise transcription and process power, while do not have coding protein ability [6,7]. Recently, fast-growing number of evidence has demonstrated that the dysregulation of lncRNA is tightly related to various diseases through involving in specific physiological and pathological processes as important regulators, such as neurological diseases [8,9]. It was first unclosed that the aberrant expression of lncRNAs was showed in SCI [10]. A study has proposed that lncRNA X-inactive specific transcript (XIST) was obviously upregulated in SCI model, and XIST decline suppressed neuron apoptosis. Therefore, XIST acted as a diagnosis and prognosis target of SCI [11]. lncRNA H19 is coded by 2.6 kb polyadenylated lncRNA, predominantly expressed in cytoplasm, and little observed in cell nucleus [12]. Ectopic lncRNA H19 expression has been found in various diseases, such as SCI [13,14,15]. After SCI, the effect of lncRNA H19 on proliferation of astrocytes has been reported lately, but the function of lncRNA H19 in neurons was not illustrated [15]. Thus, the aim of our research was to formulate the expression and function of lncRNA H19 in SCI-induced spinal neurons.

Apart from lncRNAs, microRNAs (miRNAs) serve as another one ncRNA, which have a length of 20–22 nucleotides [16]. miRNAs generally repressed the expression of proteins via binding to 3′-untranslated region of mRNA [17]. Mounting miRNAs have been reported to participate in SCI. For instance, miR-544a in SCI-injured mice was lowly expressed, and it had the potential to become a therapeutic target [18]. In SCI model, the miR-137 expression was declined, and when miR-137 was overexpressed, the SCI was recovered through hampering inflammatory and oxide stress [19]. Because miR-370-3p was predicted to be a downstream target of lncRNA H19, the influence of miR-370-3p in SCI was also explored in our study. In this research, primary spinal neuron cells were subjected to lipopolysaccharide (LPS) simulation for inducing *in vitro* injury model of SCI, and the action mechanism of lncRNA H19/miR-370-3p pathway was explored. Collectively, lncRNA H19 silencing mitigated LPS-induced spinal nerve injury through miR-370-3p upregulation, which was subjected to regulation of NF-κB signaling.

## 2 Materials and methods

### 2.1 Animal grouping

All male Sprague-Dawley (SD) rats (*n* = 12) were purchased to carry out this study. The weight of rats ranged from 250 to 300 g, and age was approximately 12 weeks. These rats were maintained under the condition of 23 ± 0.5℃ and 12/12 h light–dark cycle in a given animal room without pathogen, containing plenty of food and water. After a period of balance, rats were haphazardly assigned to two groups, namely sham group and SCI model group.


**Ethical approval:** The research related to animals’ use has been complied with all the relevant national regulations and institutional policies for the care and use of animals.

### 2.2 SCI model *in vivo*

Referring to a previous article [20], the SCI model *in vivo* was established through implementing standard T9–10 laminectomy. In short, after rats were narcotized with intraperitoneal injection of chloral hydrate (0.33 mL/kg), they were fixed on the prepared plate. Subsequently, the sterile scalpel was used for the exposure of spinal cord, and T9–10 spine was stricken to induce SCI-injured model. After the formation of SCI damage, the rats were subjected to a series of sterile anti-inflammatory treatments. Normal saline solution was used to rinse exposed spinal cord, and the wound was stitched up, as well as the rats were intraperitoneally injected with penicillin (80,000 U/0.1 mL) for 3 weeks. Bladder pressure was used to help urinate before it was possible to urinate on rat themselves. The rats in sham group were only conducted with laminectomy and without strike pressure on spinal cords.

### 2.3 Motor ability score

Motor ability is one of the main behavioral indicators. In this study, the Basso–Beattie–Bresnahan (BBB) motor was adopted to assess the motor ability of SCI rats, according to a previous reference [21]. After the establishment of SCI model, motor function was determined once a week and this experiment lasted 7 weeks. The BBB score ranged from 0 to 20 point, and 0 point represented complete paralysis and 21 point presented no injury. The final scores of BBB motor scale were obtained by three well-trained professional using the double-blind method.

### 2.4 Isolation and culture of primary spinal neurons

Primary spinal neurons were obtained to establish *in vitro* cell model. For primary spinal neurons, spinal cord tissues from SD rats were isolated and rinsed with phosphate-buffered saline (PBS, Hyclone Labs, Logan, UT, USA) and minced. The tissue mass was digested through papain (YZ-1495005, Solarbio, Beijing, China). The culture dish was pre-coated with poly-d-lysine, before primal cells were cultured originally with 10% FBS (Gibco) and 0.6% glucose (Gibco). After cultivation for 1 day, primal spinal neurons were cultivated in neural substrate medium (containing B27, GlutaMAX, and penicillin/streptomycin [Invitrogen; Thermo Fisher Scientific, Inc., Waltham, MA, USA]). The cell culture dishes were grouped in a 5% CO_2_, 37℃ incubator.

### 2.5 SCI cell model *in vitro*

For the construction of *in vitro* cell model of SCI, primary spinal neurons were stimulated with LPS. In this work, the concentration of LPS (L8880, Solarbio) was 100 ng/mL [22].

### 2.6 Reverse transcription-quantitative polymerase chain reaction (RT-qPCR)

Rat tissues and primary cells were harvested for isolation of total RNAs with TRIzol (Invitrogen). For lncRNA expression, cDNA was acquired with the PrimeScript™ RT reagent Kit (#RR037Q, Takara, China, Beijing), and the process of amplification was finished with TB Green^®^ Fast qPCR Mix (#RR430S, Takara). For the expression of miRNA, Mir-X miRNA First-Strand Synthesis Kit (#638315, Takara) was applied. The β-actin and U6 were deemed as the internal reference of lncRNA and miRNA, apart. The data were analyzed by 2^−ΔΔCt^ method.

### 2.7 3-(4,5-Dimethylthiazol-2-yl)-2,5-diphenyltetrazolium bromide (MTT)

MTT kit (M1020, Solarbio) was adopted for evaluation of cell viability. Briefly, 180 µL of cell suspension was added in plates (5 × 10^3^ cells/well, 96-well) and then cells were treated according to experimental groups. After treating the cells, the supernatant was discarded, and 90 µL of fresh culture medium and 10 µL of MTT solution were injected into every well and continuously cultivated for 4 h. Subsequently, the supernatant was discarded again and 110 µL of formazan solution was added to dissolve formazan. A microplate reader (Bio-Tek Instruments, Winooski, VT, USA) was adopted to measure optical density (OD) value at 490 nm.

### 2.8 Apoptosis assay

The Annexin V‐fluorescein isothiocyanate propidium iodide (FITC/PI) apoptosis detection kit (KeyGEN BioTECH Co. Ltd., Nanjing, China) was purchased to detect cell apoptotic rate, in light of manufacturer’s instruction. In brief, cells were collected into flow tubes and rinsed with PBS. After cells were suspended with binding buffer (500 µL), they were cultivated with Annexin V/FTIC (5 µL) and PI (5 µL) at room temperature for 15 min darkly. Cell apoptotic rate was calculated using a FACScan flow cytometer (BD Biosciences).

### 2.9 Caspase-3 activity assay

Cells cultured in 6-well plates were treated according to the experimental groups. A Caspase-3 Assay Kit (#ab39401, Abcam, Cambridge, UK) was chosen to measure the activity of caspase-3, following manufacturer’s instruction.

### 2.10 ROS generation assay

Cells bred in 6-well plates were treated according to experimental groups. A Reactive Oxygen Species (ROS) Assay Kit (Solarbio, Beijing, China) was used to determine ROS generation. Briefly, after washing with serum-free medium, cells were cultivated with DCFH-DA at room temperature for 20 min. In the end, the fluorescence intensity was tested with a microplate reader, when excitation was 504 nm and fluorescence was 529 nm.

### 2.11 Western blot

RIPA reagent (Solarbio) and BCA kit (#23235, Thermo Fisher Scientific) were chosen to conduct protein extraction and concentration quantification, several times. The different proteins of every sample were separated using gel electrophoresis and then transferred onto polyvinylidene difluoride (PVDF, Bedford, MA, USA) membranes. Then, they were covered and maintained in 5% fat-free milk at room temperature for 2 h. The primary antibodies included Bax (No. ADI-AAM-140-E, Enzo Life Sciences, Inc., Farmingdale, NY, USA), Bcl-2 (No. ADI-AAM-072-E), TNF-α (No. LS-B6067, LifeSpan BioSciences, Seattle, WA, USA), IL-6 (No. LS-C746886), IL-1β (No. 503513, San Diego, CA, USA), p-IκBα (phospho Ser32/Ser36, No. GTX79042, GeneTex, Irvine, CA, USA), t-IκBα (No. GTX27545), p-p65 (phospho Ser468, No. GTX32256), t-p65 (No. GTX107678), and β-actin (No. GTX629630). After incubation with above primary antibodies at 4℃ overnight, secondary antibodies were used to block at room temperature for 1 h. Signals of protein were developed with an ECL™ Western Blotting Analysis system (Sigma). The intensity was analyzed by ImageJ software (version 146; National Institutes of Health, Bethesda, MD, USA).

### 2.12 Luciferase reporter assays

The predicted lncRNA H19 sequence binding to miR-370-3p was amplified or mutated and inserted into the pGL3 luciferase vector (Promega, Madison, WI, USA) to obtain H19-WT or H19-MUT. The vectors carrying H19-WT or H19-MUT as well as miR-370-3p mimic or miR-NC were co-transfected into cells through Lipofectamine 2000 reagent (Invitrogen). Cells were harvested and lysed, as well as fluorescence was detected with the dual-luciferase reporter assay kit (#D0010-100T, Solarbio) to assess luciferase activity followed by the transfection of 48 h.

### 2.13 Statistical analysis

Data obtained from various experiments were analyzed by GraphPad Prism 6 (GraphPad Software, Inc., La Jolla, CA, USA) and displayed as mean ± SD. Except for comparison between the two groups, *t* test was used, and one-way ANOVA followed by *post hoc* test was used for the test. *p* < 0.05 was defined as significant difference.

## 3 Results

### 3.1 SCI-induced lncRNA H19 upregulation and miR-370-3p downregulation

SD rats were subjected to different treatment and then were assigned to SCI group and sham group. BBB scores were recorded to assess the status of rat in two groups (Figure 1a). Contrasted with sham group, the BBB scores in SCI group were dramatically reduced (*p* < 0.01, *n* = 6). Furthermore, the levels of lncRNA H19 and miR-370-3p were detected using RT-qPCR 7 days post-injury. As per the results shown in Figure 1b, it was found that lncRNA H19 was highly expressed in SCI group (*p* < 0.001) contrasted with sham group. However, miR-370-3p was downexpressed in SCI group (Figure 1c, *p* < 0.001) contrasted with sham group. The results revealed that SCI contributed to the descent of motor activity, upregulation of lncRNA H19, and downregulation of miR-370-3p.

**Figure 1:** SCI induced lncRNA H19 upregulation and miR-370-3p downregulation. After SD rats were subjected to different treatments, rats were assigned to SCI group and sham group (*n* = 6). (a) BBB scores were obtained using the double-blind method. The expression levels of (b) lncRNA H19 and (c) miR-370-3p were determined through RT-qPCR assay. *t*-test, **p < 0.01 or ***p < 0.001.

### 3.2 LPS caused spinal neuron cell injury

It has recently been shown that LPS is a major stimulus for tissue injury, resulting in inflammatory cell infiltration and necrosis of neurons in rats [23,24]. Moreover, LPS treatment was used as a stimulus in neurons or cell lines to mimic SCI *in vitro* [25,26]. In our research, primary spinal neurons were isolated from rats and stimulated with LPS for 24 h. Cell viability, apoptosis, inflammatory cytokines, and ROS generation were detected for the indication of cell injury. In Figure 2a, cell viability was significantly declined in LPS-damaged neuron cells than that in control group (*p* < 0.01). Moreover, LPS elevated cell apoptotic rate (*p* < 0.001, Figure 2b), caspase-3 activity (*p* < 0.001, Figure 2c), and Bax protein expression level (*p* < 0.001) but inhibited Bcl-2 protein level (*p* < 0.01, Figure 2d), indicating that LPS accelerated cell apoptosis. In addition, the ROS generation increase was observed in LPS-damaged cells (*p* < 0.001, Figure 2e). Furthermore, LPS treatment facilitated the protein expression of TNF-α, IL-1β, and IL-6 (all *p* < 0.001, Figure 2f). The data suggested that LPS caused spinal neuron cell injury.

**Figure 2:** LPS caused spinal neuron cell injury. Primary rat spinal neuron cells were isolated, and then spinal neuron cells were subjected to the simulation of LPS to construct SCI cell model. Untreated primary neuron cells were regarded as the control. (a) Cell viability, (b) apoptotic rate, (c) caspase-3 activity, (d) Bax and Bcl-2 protein, (e) ROS generation, (f) TNF-α, IL-1β, and IL-6 protein were examined through MTT, apoptosis, caspase-3 activity, ROS generation, and western blot assays. *t*-test. **p < 0.01 or ***p < 0.001.

### 3.3 Silence of lncRNA H19 could alleviate LPS-evoked injury

To define potential function mechanisms of lncRNA H19 during LPS-induced injury, lncRNA H19 was knocked down in spinal neuron cells via si-H19 transfection. si-H19 dramatically reduced lncRNA H19 expression compared with si-NC transfection group (*p* < 0.001, Figure 3a). After 48 h of transfection, cells were stimulated with LPS to induce SCI injury. We observed that si-H19-transfected neurons did not show an inhibition of cell viability. However, the reduction in cell viability triggered by LPS was reversed by lncRNA H19 knockdown, illustrating that silencing lncRNA H19 could alleviate LPS-declined cell viability (*p* < 0.01, Figure 3b). Furthermore, transfection of si-H19 could not aggravate spinal neuron cell apoptosis, when inducing SCI cell model through the simulation of LPS, including reduced apoptotic rate (*p* < 0.01, Figure 3c and d), caspase-3 activity (*p* < 0.01, Figure 3e) and Bax protein level (*p* < 0.01), and augmented Bcl-2 level (*p* < 0.05, Figure 3f and g), which characterized that silencing lncRNA H19 remitted LPS-induced cell apoptosis. In addition, transfecting si-H19 could not promote ROS (*p* < 0.01, Figure 3h) and above three kinds of inflammatory factor generation (all *p* < 0.01, Figure 3i and j), when inducing SCI cell model through the simulation of LPS, which unclosed that lncRNA H19 silence mitigated SCI-generated ROS and inflammatory factors. The results demonstrated that lncRNA H19 was involved in LPS-induced spinal neuron cell injury.

**Figure 3:** Silencing lncRNA H19 could alleviate LPS-evoked spinal nerve injury. (a) The si-H19 was stably transfected into spinal neuron cells to silence lncRNA H19, and lncRNA H19 expression was tested using RT-qPCR. According to different treatments, neuron cells were divided into four groups, such as control, LPS, LPS + si-NC, and LPS + si-H19 groups. (b) Cell viability, (c and d) apoptotic rate, (e) caspase-3 activity, (f and g) Bax and Bcl-2 protein, (h) ROS generation, and (i and j) TNF-α, IL-1β, and IL-6 protein were examined through MTT, apoptosis, caspase-3 activity, ROS generation, and western blot assays. One-way ANOVA analysis with Tukey’s *post hoc* test. *p < 0.05, **p < 0.01, or ***p < 0.001.

### 3.4 lncRNA H19 targeted and regulated miR-370-3p

The Starbase database was used to forecast the downstream factor of lncRNA H19. We discovered that miR-370-3p might be the downstream factor of lncRNA H19. At first, we verified above prediction that miR-370-3p acted as downstream target of lncRNA H19 using luciferase reporter assays. As shown in Figure 4a, miR-370-3p acted as the downstream target of lncRNA H19, because the luciferase activity in the group co-transfected with H19 WT and miR-370-3p was lower than that in group co-transfected with H19 WT and miR-NC (*p* < 0.001), while relative luciferase activity was not significantly different between co-transfection of H19-MUT and miR-370-3p mimic group and H19-MUT and miR-NC mimic co-transfection group (*p* > 0.05). Subsequently, the data of Figure 4b displayed that the transfection of si-H19 could contribute to miR-370-3p upregulation (*p* < 0.001). These results showed that lncRNA H19 could target and regulate miR-370-3p.

**Figure 4:** lncRNA H19 targeted and regulated miR-370-3p. (a) The predicted binding sequences between the two through Starbase database were exhibited, and then the targeted relationship between lncRNA H19 and miR-370-3p was confirmed using luciferase reporter assays. Next, we determined how lncRNA H19 regulated miR-370-3p expression. (b) The si-H19 was stably transfected into spinal neuron cells, and miR-370-3p expression was examined using RT-qPCR assay. One-way ANOVA analysis with Tukey’s *post hoc* test. ***p < 0.001.

### 3.5 Silence of lncRNA H19 could alleviate LPS-evoked injury through miR-370-3p upregulation

Therefore, we speculated that miR-370-3p was related to lncRNA H19-mediated neuron cell injury. In the following experiments, spinal neuron cells were treated with the transfection of miR-370-3p inhibitor. From the data in Figure 5a, we obtained stably transfected spinal neuron cells, as transfecting miR-370-3p inhibitor obviously declined the expression of miR-370-3p (*p* < 0.001). Besides, we also confirmed that compared with si-H19/NC inhibitor-co-transfected and LPS-induced spinal neuron cells, the viability of cell was decreased in si-H19/miR-370-3p inhibitor-co-transfected and LPS-induced cells (*p* < 0.05, Figure 5b). lncRNA H19 silence-repressed cell apoptosis was reversed through transfecting miR-370-3p inhibitor, including increased apoptotic rate (*p* < 0.01, Figure 5c and d), caspase-3 activity (*p* < 0.01, Figure 5e), and Bax protein expression (*p* < 0.01), as well as decreased Bcl-2 protein level (*p* < 0.05, Figure 5f and g). After transfection with miR-370-3p inhibitor, transfecting si-H19 could not lessen ROS generation (*p* < 0.01, Figure 5h) and inflammatory factor expression (all *p* < 0.01, Figure 5i and j). Collectively, miR-370-3p upregulation is crucial for lncRNA H19 silence to play role in SCI, and the silence of lncRNA H19 could remit LPS-induced injury through mediating miR-370-3p high expression.

**Figure 5:** The silence of lncRNA H19 could alleviate LPS-evoked spinal nerve injury through miR-370-3p upregulation. (a) miR-370-3p inhibitor was stably transfected into spinal neuron cells to silence miR-370-3p, and miR-370-3p level was tested through using RT-qPCR. According to different treatments, spinal neuron cells were divided into six groups, such as control, LPS, LPS + si-NC, LPS + si-H19, LPS + si-H19 + NC inhibitor, and LPS + si-H19 + miR-370-3p inhibitor groups. (b) Cell viability, (c and d) apoptotic rate, (e) caspase-3 activity, (f and g) Bax and Bcl-2 protein, (h) ROS generation, and (i and j) TNF-α, IL-1β, and IL-6 protein were examined through MTT, apoptosis, caspase-3 activity, ROS generation, and western blot assays. One-way ANOVA analysis with Tukey’s *post hoc* test. *p < 0.05, **p < 0.01, or ***p < 0.001.

### 3.6 Silence of lncRNA H19 could inhibit NF-κB signaling pathway through miR-370-3p upregulation

For the exploration of deep action mechanisms, NF-κB signaling pathway was excavated in this research. In Figure 6a and b, LPS fortified phosphorylation ratio of IκBα (*p* < 0.001) and p65 (*p* < 0.001). However, after transfection with si-H19, LPS-induced neuron cell did not have higher IκBα and p65 phosphorylation ratio (both *p* < 0.01). In addition, transfection of miR-370-3p inhibitor could upwardly exchange IκBα and p65 phosphorylation ratio again (both *p* < 0.01). These results suggested that silencing lncRNA H19 could inhibit NF-κB signaling through miR-370-3p mediation.

**Figure 6:** The silence of lncRNA H19 could inhibit NF-κB signaling pathway through miR-370-3p upregulation. According to different treatments, neuron cells were divided into six groups, such as control, LPS, LPS + si-NC, LPS + si-H19, LPS + si-H19 + NC inhibitor, and LPS + si-H19 + miR-370-3p inhibitor groups. (a and b) The ratio of IκBα and p65 phosphorylation was determined using western blot assay. One-way ANOVA analysis with Tukey’s *post hoc* test. **p < 0.01 or ***p < 0.001.

## 4 Discussion

SCI has a high fatality rate and the survivors are more likely to be disabled [27]. Although great efforts have been made to improve the function of SCI patients, secondary injuries by SCI are still the main cause of neurological dysfunction, characterized by neuronal apoptosis and inflammatory injury in the central nervous system [28]. Therefore, deep exploiting mechanism and avoiding apoptosis and inflammation initiation was fairly essential for SCI diagnosis and treatment. In this investigation, we found that lncRNA H19 and miR-370-3p were defined as the target of diagnosis and prognosis, thereby better stopping SCI progress from further development. To be more specific, lncRNA H19 expression was incremental and miR-370-3p was depressed in *in vivo* SCI model. There has been a study raised that LPS treats spinal neuron cell to establish *in vitro* SCI cell model [22]. The role of lncRNA H19 in SCI injury was observed that lncRNA H19 silence alleviated SCI-drove injury and blocked NF-κB signaling, which was initiated through miR-370-3p upregulation.

Aberrant lncRNA expression was defined to be the markers of diagnosis and prognosis during the occurrence and development of diseases, such as SCI. In our study, it was demonstrated that lncRNA H19 expression in SCI model was significantly different from that in sham model, and lncRNA H19 expression in SCI model was higher. In addition, silencing lncRNA H19 could mitigate LPS-caused SCI. Therefore, the upregulation of lncRNA H19 could serve as the marker of SCI diagnosis and poor prognosis. By the same token, in current researches, lncRNA H19 has already been regarded to be independent molecular target of diagnosis and prognosis in SCI [13,15]. For instance, in astrocyte post-SCI, lncRNA H19 expression was apparently raised, and the inhibition of lncRNA H19 lowered apoptosis and inflammation [15]. Moreover, the role of lncRNA H19 in a large amount of neurological diseases has also been expounded. For instance, in hypoxia/ischemia-caused neuron injury, lncRNA H19 expression level was increased, and lncRNA H19 low expression could mitigate the apoptosis of spinal neurons, thereby playing the function of protecting neurons [29]. After ischemic stroke, the lncRNA H19 level in microglial cells was elevated, and the decrease in lncRNA H19 could prevent cells from inflammatory damage [30]. In the aggregate, lncRNA H19 expression was positive in neurological diseases, such as SCI. It was potential that lncRNA H19 acted as a well-equipped biomarker in neurological diseases.

Abnormally expressed miR-370-3p has been reported in neurological disease-related researches. A glioma-associated report showed that the expression of miR-370-3p was decreased [31]. However, in cerebral aneurysm, miR-370-3p expression was augmented [32]. We also made the detection of expression level of miR-370-3p in this work, and it was observed that miR-370-3p was distinctly katabatic in SCI model. It was noteworthy that miR-370-3p was predicted to probably act as a potential downstream molecule target of lncRNA H19 through the use of Starbase database. Accumulating evidence has elucidated that lncRNAs could change some biological progress through the modulation of miRNAs in neurological diseases, such as lncRNA H19. An investigation has reported that lncRNA H19 could directly interact with miR-19a, and lncRNA H19 blockage alleviated hypoxia/ischemia-induced neuronal injury via upregulating miR-19a expression [29]. In temporal lobe epilepsy, lncRNA H19 was pronouncedly different from normal individuals, and it was overexpressed. lncRNA H19 could sponge miR-let-7b to intensify hippocampal neuron injury [33]. Besides, in astrocytes post-SCI, miR-1-3p could reverse the influence of lncRNA H19 silence in growth and activation [15]. However, in this research, it was confirmed that miR-370-3p acted as a promising downstream target of lncRNA H19 and was correlated with lncRNA H19. miR-370-3p inhibitor transfection exhibited a contrary role in LPS-induced SCI relieved by silencing lncRNA H19. Our studied results proposed the action target of lncRNA H19 in SCI process.

The activation of a number of signaling pathways has been proved to participate in cell proliferation, apoptosis, and inflammation generation, such as NF-κB pathway [34]. NF-κB acts as a lynchpin role of oncogene and the link between inflammation and cancer [35]. Furthermore, in SCI model, the NF-κB pathway was activated, and overexpressing miR-940 hampered the response of inflammation through inhibiting NF-κB pathway [36]. This result was in line with our result of NF-κB pathway in LPS-treated SCI model. LPS contributed to the activation of NF-κB pathway. There was an article that demonstrated that NF-κB signaling was mediated by ncRNAs in neurological diseases, including lncRNA and miRNA. In the article, it was found that lncRNA growth arrest-specific transcript 5 (GAS5) activated NF-κB signaling pathway and enlarged nerve cell damage via downregulation of miR-124 [37]. What is more, the regulatory effects of lncRNA H19 on NF-κB signaling pathway have been excavated in various cancers, such as human osteosarcoma [38], gastric cancer [39], melanoma [40], and glioma [41]. In cancer progression, lncRNA H19 exerted a positive function on the activation of NF-κB signaling pathway. Our results were in line with previous studied results. It was discovered that lncRNA H19 silence inactivated NF-κB signaling. Intriguingly, in present exploration, it was also monitored that lncRNA H19 silence inactivated NF-κB signaling through miR-370-3p increment. The repressed effect of miR-370-3p on this pathway was in conformity with previous study. In previous research, miR-370-3p upregulation robustly inhibited NF-κB pathway in LPS-induced *in vitro* pneumonia model [42].

To sum up, our study first testified that silencing lncRNA H19 mitigated LPS-induced neuronal injury through the mediation of miR-370-3p, which was involved in inactivation of NF-κB pathway. This study may supply novel clues for understanding the role of lncRNA H19 in SCI and offer strategies for SCI therapy.
